# LncRNA-URHC Functions as ceRNA to Regulate DNAJB9 Expression by Competitively Binding to miR-5007-3p in Hepatocellular Carcinoma

This article has been retracted.

**DOI:** 10.1155/2021/3031482

**Published:** 2021-10-07

**Authors:** Kunwei Niu, Shibin Qu, Xuan Zhang, Jimin Dai, Jianlin Wang, Ye Nie, Hong Zhang, Kaishan Tao, Wenjie Song

**Affiliations:** Department of Hepatobiliary Surgery, Xijing Hospital, Fourth Military Medical University, 127 Changle Road, Xi'an, Shaanxi 710032, China

## Abstract

**Background:**

Hepatocellular carcinoma (HCC) is often diagnosed at a late stage, when the prognosis is poor. The regulation of long noncoding RNAs (lncRNAs) plays a crucial role in HCC. However, the precise regulatory mechanisms of lncRNA signaling in HCC remain largely unknown. Our study aims to investigate the underlying mechanisms of lncRNA (upregulated in hepatocellular carcinoma) URHC in HCC.

**Objective:**

To study the in vivo and in vitro localization and biological effects of URHC on liver cancer cells. Through bioinformatics analysis, dual-luciferase reporter gene analysis and rescue experiments revealed the possible mechanism of URHC.

**Methods:**

RT-qPCR, fluorescence in situ hybridization (FISH) staining, EdU, colony formation, and tumor xenograft experiments were used to identify localized and biological effects of URHC on HCC cells in vitro and in vivo. The bioinformatics analysis, dual-luciferase reporter assay, and rescue experiments revealed the potential mechanism of URHC.

**Results:**

URHC silencing may inhibit the HCC cells' proliferation in vitro and in vivo. We found that URHC was mainly localized in the cytoplasm. The expression of miR-5007-3p was negatively regulated by URHC. And miR-5007-3p could reverse the effect of URHC in HCC cells. The expression of DNAJB9 was negatively regulated by miR-5007-3p but positively regulated by URHC. These suggestive of lncRNA-URHC positively regulated the level of DNAJB9 by sponging miR-5007-3p.

**Conclusion:**

Together, our study elucidated the role of URHC as a miRNA sponge in HCC and shed new light on lncRNA-directed diagnostics and therapeutics in HCC.

## 1. Introduction

Hepatocellular carcinoma (HCC) is the most common type of liver tumor worldwide. It has become the second leading cause of cancer-related death in China [1, 2]. Tumor resection is currently the best treatment choice among the several therapeutic methods available. However, HCC is often diagnosed at a late stage when the rupture of HCC caused haemoperitoneum, which is with poor prognosis generally [3]. The extrahepatic metastases of HCC represent a poor prognostic factor. In particular, orbital metastasis rarely occurs [4]; and many patients die within 1 year after the detection of HCC [5]. Therefore, enhancing our understanding of the molecular mechanisms in HCC is essential for the development of effective treatment strategies. Recent experimental studies provide strong evidence that lncRNAs play an important role in cancer progression, and the abnormal expression of lncRNAs has been found in the HCC [6–9]. For example, lncRNA HOST2 can activate the JAK2-STAT3 signaling pathway and promote epithelial-mesenchymal transition, proliferation, invasion, and migration of HCC cells [9]. A lncRNA PVT1/miR-150/HIG2 axis regulates the proliferation, invasion, and balance of iron metabolism in HCC [10]. LncRNAs have been shown to function as miRNA sponges, which interact with miRNAs and play crucial roles in human carcinogenesis by modulating the expression of miRNA target genes [11–14]. These may contribute to the development of new effective therapeutic strategies to improve the prognosis of HCC patients.

Many aberrant expression patterns of lncRNAs have been found to be associated with human diseases, in particular, cancers [15–19]. They can regulate gene expression in cis or in trans by diverse mechanisms [20–22] and have been demonstrated to cause dysregulation of lncRNAs and impact on cellular functions such as cell proliferation, apoptosis, migration, invasion, tumorigenicity, and metastasis, by interacting with DNA, RNA, and proteins [23, 24]. By negatively regulating the expression of target genes, miRNAs play a significant role at the posttranscriptional level and participate in a large number of biological processes, including cell proliferation, cell cycle, apoptosis, and differentiation [25–29]. Recent studies have revealed that lncRNAs can function as competing endogenous RNAs (ceRNAs) to regulate the expression pattern and biological characteristics of miRNAs [30, 31].

In the present study, we investigated the biological effects of URHC overexpression on cell proliferation in HCC. Bioinformatics prediction and experimental analysis confirmed that URHC directly targeted miR-5007-3p to regulate its expression. Furthermore, mechanistic analysis revealed that URHC positively regulated DNAJB9 by sponging miR-5007-3p, indicating that it plays an oncogenic role in HCC pathogenesis. Together, these results suggest that the molecular mechanisms of URHC-miR-5007-3p-DNAJB9 axis are likely to be enriched in HCC.

## 2. Materials and Methods

### 2.1. Cell Culture and Transfection

The human HCC cell line Hep3B and 293T cells were purchased from ATCC. The normal human liver cell line MIHA was purchased from YaJi Biological (Shanghai, China). HCC cells Bel-7402 and Bel-7404 were obtained from Beina Biological (Beijing, China) in 2017. The SMMC-7721 was bought from Fenghui Biotechnologies Inc. (Hunan, China). MIHA, SMMC-7721, Bel-7402, and Bel-7404 cells were cultured in RPMI 1640 (Invitrogen, Carlsbad, CA, USA) containing 10% fetal bovine serum (FBS, Invitrogen). Hep3B and 293T were cultured in Dulbecco's modified Eagle medium (DMEM, Invitrogen) containing 10% FBS. All cells were incubated in a humidified atmosphere of 5% CO_2_ at 37°C. Dimethyl sulfoxide was purchased from Sigma-Aldrich (St. Louis, MO).

Scrambled siRNA of URHC (siRNA-Con) and URHC siRNAs were purchased from GenePharma (Shanghai, China). miR-5007-3p inhibitor, inhibitor negative control (NC inhibitor), miR-5007-3p mimic, and NC mimic were also purchased from GenePharma (Shanghai, China). Full-length URHC cDNA was subcloned into GV230 lentiviruses (Genechem, Shanghai, China) and infected into Bel-7404 and Hep3B cells to generate URHC-overexpressing cells. Lipofectamine 2000 Reagents (Invitrogen Co., USA) were used for cell transfections.

### 2.2. Human Tissue Samples

We obtained 26 pairs of primary HCC and adjacent nontumor tissues from patients undergoing surgery at Xijing Hospital, the Fourth Military Medical University; all diagnoses were based on a biopsy. These tissues were immediately frozen in liquid nitrogen after surgical resection. All patients provided written informed consent, and these studies were approved by the Ethics Review Committees of Xijing Hospital.

### 2.3. Reverse Transcription and Quantitative Real-Time PCR

Total RNA was prepared from the indicated cells using TRIzol reagent (Invitrogen) based on the manufacturer's instructions. One microgram of total RNA was converted to cDNA using PrimeScript® RT Master Mix Perfect Real-Time (Takara, Inc). SYBR Premix EX Taq II (TaKaRa) was used based on the manufacturer's instructions under the following conditions: 95°C for 2 min, 95°C for 15 s, and 60°C for 60 s for 40 cycles. miR-5007-3p expression levels were quantified using MicroRNA First-Strand Synthesis and miRNA Quantitation Kits including U6 control primer (Takara) based on the manufacturer's instructions. The results were analyzed based on the 2^−ΔΔCT^ formula [32]. The primers used for RT-qPCR were as follows: *β*-actin: sense 5′-CTGGAACGGTGAAGGTGACA-3′, and antisense 5′- CGGCCACATTGTGAACTTTG-3′; URHC: sense 5′- TGTTTATGTGAGAGGAGAAAGGAAG-3′; and antisense 5′- CACTAGAGGTCTGCAAATAAAGTGA-3′; DNAJB9: sense 5′- TAGGCACACACCACCACATC-3′; and antisense 5′- CTTTGGGAGGCCAAGGTAGG-3′; and miR-5007-3p 5′-CCATATGAACCAAACTCTAATA-3′. The internal control genes were *β*-actin for URHC, DNAJB9, and U6 snRNA for miR-5007-3p.

### 2.4. Fluorescence In Situ Hybridization

SMMC-7721 and Hep3B cells were plated to achieve 70% confluency for staining. Frozen sections of HCC tissues were treated with 4% DNase/RNase-free paraformaldehyde. After fixation, the sections were treated with Proteinase K (20 g/ml) for 5 min and then washed three times with phosphate-buffered saline (PBS). The cells were incubated with a prehybridization solution for 1 h at 37°C. Then, the prehybridization solution was removed, and the cells were covered with a URHC probe (8 ng/*μ*l) hybridization solution overnight in a 37°C incubator. The slices were washed three times using Wash Buffer Solution. The cells were extensively washed three times using Wash Buffer Solution, counterstained with DAPI, and mounted with an antifade reagent (Invitrogen). The URHC probe for fluorescence in situ hybridization (FISH) was 5′-GFP-AGTACATACTCACTACACTAGAGGTCTGCA-GFP-3′ (Servicebio, China). The mir-5007-3p probe for FISH was 5′-Cy3-ATTAGAGTTTGGTTCATATGAT-Cy3-3′ (Servicebio).

### 2.5. CCK-8 and Colony Formation Assays

The CCK-8 assay was used to assess HCC cell proliferation. HCC cells were seeded in a 96-well plate at a density of 2 × 10^3^ cells per well. Cell proliferation was measured at 24, 48, 72, and 96 h. CCK-8 solution (10 L) was added to each well, and incubated for 1 h at 37°C, in a 5% CO_2_ incubator. After incubation, the optical density (OD) 450 value was read using an Epoch Spectrophotometer (USA). Experiments were repeated at least three times.

The colony formation assay was performed to measure the capacity of cell proliferation. SMMC-7721 and Hep3B cells (300 cells/well) were seeded in a six-well plate and cultured for 10 days. Colonies were then fixed with methanol for 15 min and stained for 10 min with 0.5% crystal violet. Then, colonies were imaged with a phone and analyzed by ImageJ software. The assays were repeated at least three times.

### 2.6. 5-Ethynyl-2′-Deoxyuridine (EdU) Assay

Cell proliferation was also determined by the 5-ethynyl-2′-deoxyuridine assay using an Apollo®488 EdU Kit (RIBOBIO, Guangzhou, China). The EdU assay was performed based on the manufacturer's instructions. The cells were then visualized under a fluorescence microscope (20 × 10). To assess cell proliferation, the ratio of EdU-stained cells (with red fluorescence) to Hoechst-stained cells (with blue fluorescence) was calculated. Experiments were repeated at least three times.

### 2.7. Luciferase Reporter Assay

The luciferase reporter assay was performed in 293T cells. The 293T cells were seeded in a six-well plate and cotransfected with luciferase reporter constructs encoding the wild-type 3′-UTR region of DNAJB9 or URHC (DNAJB9/URHC-WT-3′-UTR) or a mutated 3′-UTR region of DNAJB9 or URHC 3′-UTR region (DNAJB9/URHC-MUT-3′-UTR) (RIBOBIO, Guangzhou, P.R. China) and miR-5007-3p mimic or mi-NC using Lipofectamine 2000 (Invitrogen). After 48 h of incubation, the cells were washed with PBS and lysed with Passive Lysis Buffer (Promega). Firefly and Renilla luciferase activities were measured using the dual-luciferase reporter assay kit (Promega) based on the manufacturer's protocol.

### 2.8. Western Blot Assay

Cells were lysed using RAPI buffer (Beytime, China). Total proteins were quantified using the BCA Protein Assay Kit (Beytime, China). Proteins were separated by 12% SDS-polyacrylamide gel electrophoresis and transferred to a polyvinylidene fluoride (PVDF) membranes (Milipore, Inc.). The membranes were washed three times for 10 mins with Tris-buffered saline-0.5% Tween 20 (TBS-T) and blocked with 5% nonfat milk-TBS-T at room temperature for 1 h. Subsequently, they were incubated with primary antibodies (anti-DNAJB9 (1 : 1000) and anti-GAPDH (1 : 1000) obtained from Abcam and Cell Signaling Technology, respectively) at 4°C overnight. Following incubation with corresponding secondary antibodies, the signals were detected with ECL Western Blotting Detection Reagents (Milipore, Inc.). GAPDH was used as an endogenous reference.

### 2.9. Immunohistochemical (IHC) Assay

DNAJB9 and Ki67 were detected in xenograft tumor specimens of nude mice, which were fixed with paraformaldehyde, embedded with paraffin, and cut into 4 *μ*m sections. The subsequent steps accomplished with the biotin-streptavidin peroxidase method (SPlink Detection Kit, ZSGB-Bio, Beijing, China) were followed based on the manufacturer's instructions. Briefly, paraffin-embedded samples were deparaffinized, dehydrated in a graded series of ethanol and blocked with endogenous peroxidase for 10 min, and incubated in goat serum for 30 min. The slides were incubated with the corresponding primary antibodies at 4°C overnight. Then, the slides were washed with PBS, incubated with biotinylated goat anti-rabbit IgG, and then incubated with horseradish peroxidase (HRP) conjugated streptomycin. Diaminobenzidine (ZSGB-Bio) was added to the slides for chromogenic reaction. The slides were observed with an optical microscope (Olympus, Tokyo, Japan).

### 2.10. In Vivo Proliferation Assay

Six-week-old male BALB/c nude mice were obtained from Vital River Laboratory Animal Technology Co. (Beijing, China). Animal studies were approved by the Institutional Animal Care and Use Committee of Fourth Military Medical University. The mice were housed in pathogen-free conditions. To further determine the antitumorigenesis potential of URHC in vivo, 7721 cells transfected with siRNA-NC and URHC-siRNA were inoculated into male nude mice. Mice were randomly divided into two groups with five mice in each group, but each group only included three tumors. siRNA-URHC and URHC-NC cells (1 × 10^7^) were inoculated subcutaneously in the right flank of nude mice. Tumors were measured every 7 days, and tumor volumes were calculated. Five weeks after HCC cell inoculation, the mice were sacrificed, and the tumors were collected.

### 2.11. Statistical Analysis

All experimental data were reported as means ± experimental standard deviations (SD). Student's *t*-test was used to determine the significance of the results (significance: ^*∗*^*P* < 0.05;  ^*∗∗*^*P* < 0.01;  ^*∗∗∗*^*P* < 0.001).

## 3. Results

### 3.1. URHC Promotes Cell Proliferation of HCC In Vitro and In Vivo

Previous data indicate that URHC expression is upregulated in HCC cell lines and tissues [33]. 7404 and Hep3B cells exhibited lower URHC expression than the 7721 and 7402 HCC cell lines (Figure 1(a)), so we selected 7404 and Hep3B cells to construct stable cell lines to overexpression URHC, and the transfection efficiency was detected by RT-qPCR (Figure 1(b)). The previous results of CCK-8 and EdU assays demonstrated that the downregulated expression of URHC attenuated the proliferation of 7721 cells [32], whereas the overexpression of URHC enhanced 7404 and Hep3B cells proliferation by CCK-8 and colony formation assays (Figures 1(c) and 1(d)). Mice injected with siRNA-URHC 7721 cells showed a reduction in tumor volume and weight at the end of the experiment compared with the control groups (Figures 1(e)–1(g)). Moreover, IHC staining revealed that Ki67 (proliferation marker) expression was decreased in the siRNA-URHC xenograft tumor tissues (Figure 1(h)). These results suggest that URHC expression may play an important role in the cell proliferation of HCC in vitro and in vivo.

### 3.2. URHC Is Predominantly Localized in the Cell Cytoplasm

Since many lncRNA are not restricted to either the nuclear or cytoplasmic compartment [34, 35], but cellular location is known to dictate the function of lncRNAs. However, the subcellular location of URHC is unclear. A FISH assay was performed to identify the subcellular localization of URHC in 7721 cells, Hep3B cells, HCC tissues, and adjacent tissues. Moreover, cellular fractionation was performed to identify the subcellular localization of URHC in 7721 and Hep3B cells. The results confirmed that URHC was mainly localized in the cell cytoplasm (Figures 2(a)–2(c)).

### 3.3. URHC Can Function as ceRNA to Sponge miR-5007-3p

Increasing evidence has revealed that lncRNAs contain sequences that are complementary to miRNAs and that they can directly or indirectly regulate the expression and activity of miRNAs. The potential targets of URHC were predicted by the bioinformatics database (StarBase). We observed that several potential miRNAs had putative binding sites for URHC, such as miR-5007-3p, miR-4698, miR-559, and miR-3942-3p (Table 1). Compared with the other three potential miRNAs, the expression level of miR-5007-3p was the lowest in the URHC high expressing of HCC cells and highest in the URHC low expressing HCC cells (Figures 3(a) and S1). Next, we measured the expression of miR-5007-3p in HCC tissues and normal tissues. As shown in the RT-qPCR results in Figure 3(b), the expression of miR-5007-3p was significantly downregulated in HCC tissues compared with that in the adjacent tissues. To confirm our prediction that miR-5007-3p targets URHC, we first measured the expression levels of miR-5007-3p in 7404, Hep3B, 7721, and 7402 cells that were transfected with over-URHC or siRNA-URHC, respectively, by RT-qPCR. The results showed that the expression of miR-5007-3p was decreased in the over-URHC group compared with the overcontrol group, whereas the expression of miR-5007-3p was increased in the siRNA-URHC group compared with the siRNA-control group (Figure 3(c)). Meanwhile, RT-qPCR analysis of resected tumor tissues demonstrated same results (Figure 3(d)). Additionally, we determined the location of URHC and miRNA-5007-3p in HCC tissues, normal tissues, and cell lines. The FISH results showed that URHC and miRNA-5007-3p were colocalized in the cell cytoplasm (Figure 3(e)). These results suggest that URHC may negatively regulate the expression of miR-5007-3p. Moreover, we confirmed the direct relationship between URHC and miR-5007-3p using a dual-luciferase reporter assay. Using the bioinformatic database, we predicted the potential miRNA binding sites in URHC, and the alignment of miR-5007-3p with the 3′-UTR of URHC was shown (Figure 3(f)). 293T cells were cotransfected with miRNAs and URHC (URHC-NC, URHC mutant). As shown in Figure 3(g), miR-5007-3p mimic transfection significantly decreased the luciferase activities of URHC compared with NC transfection, whereas there were no effects on the luciferase activities by miR-5007-3p mutant transfection. These results indicate that URHC directly targets miR-5007-3p to regulate its expression.

### 3.4. miR-5007-3p Reverses the Promoting Effect of URHC on Cell Growth

We next determined whether URHC exerted its function through miR-5007-3p in 7721 and Hep3B cells in EdU and colony formation assays. The proliferation of 7721 cells in the siRNA-URHC + miR-5007-3p inhibitor group was remarkably increased compared with that in the siRNA-URHC and siRNA-URHC significant + miR-5007-3p inhibitor NC groups, whereas HCC cell proliferation was evidently decreased in the over-URHC + miR-5007-3p mimic group compared with the over-URHC and over-URHC + miR-5007-3p mimic NC groups (Figures 4(a) and 4(b)). These results suggest that URHC function was reversed by transfection with miR-5007-3p inhibitor or mimic in 7721 and Hep3B cells.

### 3.5. URHC Regulates the Expression of DNAJB9 by Targeting miR-5007-3p in HCC Cells

It is well known that miRNAs play biological roles by targeting the 3′-UTR of target genes. The bioinformatics databases (miRDB, miRTarBase, and miRWalk) predicted that potential downstream genes of miR-5007-3p include BCOR, AJAP1, DNAJB9, RAI1, and others (Figures S2A and S2B). Among the targets of miR-5007-3p, we focused on DNAJB9, because the expression level of DNAJB9 was the highest in the HCC cells that highly expressed URHC (Figure S2C). We first measured the expression of DNAJB9 in HCC tissues, and its expression was found to be significantly increased (Figure 5(a)). In 7721 and 7402 cell lines, the mRNA level of DNAJB9 was significantly decreased in cells transfected with siRNA-URHC compared with control cells, whereas the expression of DNAJB9 in over-URHC cells showed the opposite result (Figure 5(b)). Meanwhile, RT-qPCR and Western blot analysis of resected tumor tissues demonstrated DNAJB9 was decreased in the siRNA-URHC group compared with the siRNA-control group (Figures 5(c) and 5(d)). Furthermore, the URHC and DNAJB9 expression showed a significant positive correlation in HCC patients by Spearman's correlation analysis, whereas miR-5007-3p and DNAJB9 expression showed a significant negative correlation (Figure 5(e)). Using the bioinformatic database, we predicted the potential miRNA binding sites in DNAJB9, and the alignment of miR-5007-3p with the 3′-UTR of DNAJB9 was shown (Figure 5(f)). We then confirmed the direct interaction between miR-5007-3p and the 3′-UTR of DNAJB9 using a dual-luciferase reporter assay. 293T cells were cotransfected with miRNAs and DNAJB9 (DNAJB9 NC, DNAJB9 mutant). As shown in Figure 5(g), miR-5007-3p transfection significantly decreased the luciferase activities of DNAJB9, compared with NC transfection, whereas there were no effects on the luciferase activities by miR-5007-3p mutant transfection. Furthermore, we determined whether miR-5007-3p was involved in the URHC regulation of DNAJB9 expression. We assessed the effects of URHC and miR-5007-3p on the mRNA and protein levels of DNAJB9 by RT-qPCR and Western blot and found that DNAJB9 expression levels were apparently affected by URHC and miR-5007-3p. As shown in Figures 5(h) and 5(i), DNAJB9 expression was significantly decreased after transfecting with siRNA-URHC and miR-5007-3p inhibitor NC. The inhibitory effect of siRNA-URHC was notably reversed by cotransfection with siRNA-URHC and miR-5007-3p inhibitor in 7721 cells. Otherwise, the expression of DNAJB9 was significantly increased in the over-URHC and miR-5007-3p mimic NC groups. The above results suggested that URHC functioned as a ceRNA by sponging miR-5007-3p and indirectly regulated DNAJB9 expression.

## 4. Discussion

In this study, we added the function of URHC in vivo and in vitro. URHC is predominantly in the cell cytoplasm and this indicates that URHC can function as ceRNAs to regulate the expression pattern and biological characteristics of miRNAs. Our study showed URHC high expression in HCC tissues and cell lines, while miR-5007-3p is low expression. In addition, miR-5007-3p can reverse the promoting effect of URHC on cell growth. However, URHC promotes cell proliferation of HCC and inhibiter miR-5007-3p is by regulation downstream DNAJB9. The study highlights the role of URHC in HCC and highlights URHC as a potential diagnostic and therapeutic target.

LncRNAs were upregulated in hepatocellular carcinoma (URHC), and our research group screened for a novel lncRNA. It is located on the forward strand of human chromosome 2 : 173958088–173958307, and its transcript length is 219 bp. The previous result shows that it was highly expressed in HCC cell lines, clinical HCC tissues, and poor survival in HCC patients, and URHC high expression promoted tumor growth and inhibited apoptosis via ERK/MAPK inactivation by targeting ZAK [33]. However, the precise regulatory mechanisms of URHC signaling in HCC are still largely unknown. In this study, we investigated the expression pattern of URHC in HCC. The results confirmed that URHC was preferentially localized in the cell cytoplasm, suggesting that it could function as a ceRNA to regulate the expression pattern and biological characteristics of miRNAs.

Many miRNAs have been shown to play a regulatory role in HCC, regulating the biological behavior of HCC cells, thereby affecting tumor progression. A study has shown that miR-5007-3p is expressed in the lymphatic metastasis tissue from gastric cancer patients via RT-qPCR. In addition, the results revealed that expressed of miR-5007-3p was upreglated in patients with positive lymphatic metastasis of primary gastric tumors [36]. In addition, another experiment by RT-qPCR indicated that the relative expression level of miR-5007-3p was significantly upregulated in the diabetic kidney disease group compared to type 2 diabetes group [37]. However, these researches did not examine miR-5007-3p specific cellular functions, and miR-5007-3p expression in HCC is unclear. Whether the important roles of URHC in HCC are associated with the dysregulation of miR-5007-3p also remains unknown. In our study, we found that the expression level of miR-5007-3p was the lowest in the URHC high expressing HCC cells and highest in the URHC-low expressing HCC cells, an inverse correlation between URHC and miR-5007-3p expression. And miR-5007-3p could reverse the promoting effect of URHC on cell proliferation.

DNAJ homolog subfamily B member 9 (DNAJB9), also known as MDJ-1 and ERDJ4, is a 223-amino acid protein that is a member of the DNAJ protein family [38]. The research shows that it is expressed in most cells and displays cytoplasmic immunoreactivity, and DNAJB9 is an unique ER luminal cochaperone that may involve a pair of chaperones from the cytosol and the ER [39, 40]. Moreover, the study reported that DNAJB9 is involved in ER stress and in the unfolded protein response (UPR) and can inhibit IRE1 activation and degrade SREBP1c, thereby reducing insulin resistance and tumorigenesis in mTORC1/2 constitutively active mice [41]. Another ability of DNAJB9 is to promote liver hypertrophy and suppress food intake. Meanwhile, DNAJB9 influences many cellular processes by regulating the ATPase activity of 70 kD heat shock proteins [38, 42]. However, the cellular function of this DNAJB9 remains largely unknown. Our results showed that URHC bound directly to miR-5007-3p, thereby controlling miR-5007-3p availability for its target gene DNAJB9. Furthermore, we confirmed that DNAJB9 was highly associated with URHC.

## 5. Conclusion

In summary, URHC promoted HCC cell proliferation in vitro and in vivo, suggesting that URHC exhibited oncogenic properties in HCC progression. URHC promoted proliferation via sponging miR-5007-3p from DNAJB9 both in vitro and in viv*o*. Due to time and funding issues, more regulatory mechanisms and target genes have not been studied, but this URHC/miR-5007-3p/DNAJB9 regulatory network may help clarify tumorigenesis in HCC and may help to develop new diagnosis and treatment methods for HCC.

## Figures and Tables

**Figure 1:** URHC promotes cell proliferation of HCC in vitro and in vivo. (a) Relative expression of URHC was detected by qRT-PCR in HCC cell lines. (b) Increased expression of URHC was detected using RT-qPCR. (c) 7404 and Hep3B cells were stably transfected with over-URHC or overcontrol, and cell viability was measured using the CCK-8 assay at 24, 48, 72, and 96 h. (d) Colony formation assay in 7404 and Hep3B cells stably transfected with over-URHC or overcontrol. (e) Xenograft tumors from the nude mice are shown. Each group contained five nude mice. (f) Tumor growth curves were analyzed. (g) Tumor weights were analyzed. (h) Immunohistochemistry analysis of Ki-67 was obtained from tumors. Magnification: ×400.

**Figure 2:** The subcellular location of URHC in HCC cell lines and tissues. (a) Detection of URHC by fluorescence in situ hybridization (FISH) in HCC cell lines 7721 and Hep3B. URHC: endogenous URHC; DAPI: DNA stained with DAPI; merge: merged images of DAPI and URHC immunofluorescence. Magnification: ×400. (b) FISH was performed to analyze URHC in HCC tissues and adjacent tissues. Magnification: ×400. (c) Cellular localization of URHC in 7721 and Hep3B cells is shown. GAPDH and U6 served as a cytoplasmic and nuclear localization marker, respectively. ^*∗*^*P* < 0.05.

**Figure 3:** URHC was a target of miR-5007-3p. (a) Relative expression of miR-5007-3p in HCC cell lines and normal hepatic cells was detected by qRT-PCR. (b) Relative expression of miR-5007-3p in HCC tissues and adjacent tissues was detected by qRT-PCR. (c) RT-qPCR analysis of URHC-regulated miR-5007-3p expression in 7721, 7402, 7404, and Hep3B cells. (d) The expression level of miR-5007-3p in tumors was detected. (e) FISH was performed to analyze the colocalization of URHC and miR-5007-3p in HCC cell lines and tissues. Magnification: ×400. (f) The predicted miR-5007-3p binding sites in URHC-WT and the designed mutant sequence (URHC-MUT) were indicated. (g) Luciferase reporter assay of 293T cells cotransfected with URHC-WT or URHC-MUT and miR-5007-3p NC or miR-5007-3p. The bars represent means ± SD of three independent experiments.  ^*∗∗*^*P* < 0.05,  ^*∗∗*^*P* < 0.01, and  ^*∗∗∗*^*P* < 0.001 compared with the control group.

**Figure 4:** miR-5007-3p reversed the promoting effect of URHC on the growth of HCC cells. (a, b) EdU and colony formation assays identified the phenomenon of URHC regulating each other to compete for the binding of miR-5007-3p in 7721 and Hep3B cell lines. Magnification: ×400.

**Figure 5:** URHC regulated the expression of DNAJB9, an endogenous miR-5007-3p target. (a) Relative expression of DNAJB9 in HCC tissues and adjacent tissues was detected by qRT-PCR. (b) RT-qPCR analysis of URHC-regulated DNAJB9 expression in 7721, 7402, 7404, and Hep3B cells. (c, d) The mRNA and protein levels of DNAJB9 in tumors were assessed. (e) The positive correlation between URHC and miR-5007-3p expression and the negative correlation between miR-5007-3p and DNAJB9 expression in HCC tissues are shown in scatter diagrams. (f) The predicted binding sites of miR-5007-3p in the DNAJB9 sequence are shown. (g) Luciferase reporter assay of 293T cells cotransfected with DNAJB9-WT or DNAJB9-MUT and miR-5007-3p NC or miR-5007-3p. (h, i) The levels of DNAJB9 in HCC cells transfected with miR-5007-3p inhibitor/mimic or siRNA-URHC/over-URHC were analyzed by RT-qPCR and western blot. ^*∗*^*P* < 0.05,  ^*∗∗*^*P* < 0.01, and  ^*∗∗∗*^*P* < 0.001.

**Table 1:** StarBase online predicted miRNAs that target URHC.

Name	Accession	Query start	Query start	Subject start	Subject end	Score	Evalue
Has-miR-5007-3p	MIMAT0021036	74	91	4	21	72	1.5
Has-miR-4698	MIMAT0019793	59	73	2	16	66	4.7
Has-miR-559	MIMAT0003223	66	85	1	20	64	6.9
Has-miR-3942-3p	MIMAT0019230	164	181	4	21	63	8.3

## Data Availability

The data used to support the findings of this study can be obtained from the corresponding author upon reasonable request. Additional supporting information may be found online in the Supplementary Materials section.

## Supplementary Materials

Supplementary Materials Figure S1: RT-qPCR analysis for URHC-regulated miR-5007-3p, miR-559, miR-3942-3p, and miR-4986 expression in 7721, 7402, 7404, and Hep3B cells. ^*∗*^*P* < 0.05,  ^*∗∗*^*P* < 0.01, and  ^*∗∗∗*^*P* < 0.001. Figure S2: (A, B) miRDB, miRTarBase, and miRWalk predicted some of the RNAs targeted by miR-5007-3p. (C) RT-qPCR analysis for URHC regulated the expression of an endogenous miR-5007-3p target gene (BCOR, AJAP1, DNAJB9, RAI1, ZNF711, DDT, and WDR35) in HCC cells (Huh7, HepG2, 7402, 7721, SNU368, 7404, and Hep3B) and normal human hepatocyte cell line MIHA. ^*∗*^*P* < 0.05,  ^*∗∗*^*P* < 0.01, and  ^*∗∗∗*^*P* < 0.001.
